This article has been retracted.

# Application of Artificial Intelligence Computing in the Universal Design of Aging and Healthy Housing

**DOI:** 10.1155/2022/4576397

**Published:** 2022-03-26

**Authors:** Quanfa Shu, Hui Liu

**Affiliations:** ^1^Shenzhen Grandland Building Decoration Design Institute, Shenzhen, Guangdong 518003, China; ^2^Graduate School, Hoseo University, Asan, Chungcheongnam-do 31499, Republic of Korea; ^3^Zhengzhou Business University, Zhengzhou, Henan 451200, China

## Abstract

Intelligent control technology is not only the use of the so-called highly sophisticated technology in the daily life of the elderly but also control services according to the individual needs of the elderly. This paper combines research in psychology and ergonomics to explore how to use the living space to build indoor scenarios that influence the behavioural and psychological changes of the elderly based on satisfying functionality. The external environment influences the user's perception, and the perception determines the user's behaviour. Through the construction of scenarios, objects and people can interact with each other, thus achieving the objective of “solitude but not loneliness” for the elderly living alone and providing a modern ageing environment with high safety, convenience, quality, and comfort for the elderly.

## 1. Introduction

With the development of ageing population, developed countries such as Europe and the United States are entering an ageing society first. More and more attention is being paid to the issue of elderly people's retirement. With their strong economic strength and the advantages of science and technology, developed countries have been developing their medical and healthcare services. Especially with the rapid development of electronic and information technology, developed countries have taken the lead in exploring the use of information technology to help traditional elderly care [1]. After IBM put forward the concept of “smart city,” countries such as the UK, the US, and Japan have also put forward the concept of “intelligent old-age care” or “intelligent care for ageing.” The market-oriented operational characteristics of smart old-age care in developed countries are obvious, and the degree of commercialisation is high [2].

Commercial enterprises carefully analyse the needs of the elderly for elderly care services, constantly optimise user experience, and apply new technologies, so as to develop newer and better products for smart elderly care services, including health and medical information sharing data platforms for the elderly, smart elderly community management platforms, emergency call systems, and intelligent elderly care terminal products. A theoretical system and industrial chain for smart elderly care have been initially formed [3].

Old and frail, with children at home, but living alone in a small space or courtyard bungalow is the current situation of the elderly living alone in China. They are relatively capable of taking care of themselves, but can only maintain the status quo for the time being. As they grow old and live alone in small space for long periods of time and rarely leave their homes, they gradually become isolated from their neighbours and society and have a great need for spiritual comfort. The elderly long for companionship, but their families cannot be there for long.

Every family has an elderly person, but not every elderly person has a family member with them. It is easier to know than to do. At least one-third of urban families are of the empty nest type, that is, elderly people living alone or an elderly couple with no children. While paying more attention to these elderly people, the research aims to address the loneliness of the elderly living alone, improve the quality of their lives and living environment, and meet their physical and mental needs through scenario-based design so that they do not feel lonely even when living alone. The study aims to improve the quality of the elderly's living and living environment through scenario-based design, so that they do not feel lonely even when living alone [4].

China has also entered a phase of rapid population ageing. On the whole, the problem of insufficient supply of elderly services and products and the structural imbalance in the supply of social elderly service resources is also becoming increasingly prominent. Taking advantage of the opportunities brought about by the rapid development of the Internet and information technology, it has become an important task to build a well-off society to resolve the contradiction between the growing demand for elderly services and the unbalanced and insufficient development. Compared with developed countries, China is relatively late in the process of population ageing, and the development of the domestic smart elderly care industry is still in the initial exploration stage. Therefore, by comparing and studying the smart ageing in developed countries such as Europe, America, and East Asia and then combining the actual situation of ageing in China, summarising the experience suitable for the development of smart ageing in China will help to build and improve a smart ageing service system with Chinese characteristics [5].

The birth of intelligent device control technology is the result of the mutual reaction between the pursuit of high-quality physical and mental health of the elderly and the rapid development of information technology. Intelligent control technology is not only the use of the so-called highly sophisticated technology in the daily life of the elderly but also control services according to the individual needs of the elderly. This paper combines research in psychology and ergonomics to explore how to use the living space to build indoor scenarios that influence the behavioural and psychological changes of the elderly based on satisfying functionality. The external environment influences the user's perception, and the perception determines the user's behaviour. Through the construction of scenarios, objects and people can interact with each other, thus achieving the objective of “solitude but not loneliness” for the elderly living alone and providing a modern ageing environment with high safety, convenience, quality, and comfort for the elderly.

## 2. Related Work

Many efforts have relied on existing Internet resources and social forces to build public information platforms and senior care information service network platforms using technologies such as cloud computing and big data to provide community-based care and nursing, health management, rehabilitation, and other home care services. For example, the authors of [6] proposed the concept of “digital community” and “digital elderly care” and conducted research and discussion. The authors of [7] introduced the Hangzhou digital community to realize the livelihood project of “digital elderly care” in the district. Söker et al. [8] proposed a networked home care model. Ostrowski [9] proposed a strategy for the construction of digital elderly care services in the context of new urbanisation. The authors of [10] put forward the concept of smart elderly care, pointing out that smart elderly care is the use of the Internet of Things, cloud computing, and other technologies to carry out comprehensive, online and offline, integrated medical care and all-round elderly care services. Glavič et al. [11] emphasised that smart ageing provides comprehensive services for the elderly in terms of clothing, food, housing, transport, entertainment, and health, helping them to improve their quality of life while not forgetting to help them reflect their value and dignity. The authors of [12] argued that smart ageing is a new model of elderly care services, the core of which lies in taking the needs of the elderly in groups as the guide, mobilising various elderly care resources to coordinate the actions of various elderly care-related parties through the integration of advanced management and information technology, so as to systematically, intelligently, and humanely improve the capacity and level of community elderly care services at home, and strive to provide the lowest cost, highest efficiency, and most convenient services, solving the problem of ageing in place for the elderly in the community.

In response to the characteristics of the scattered population living in the United States, a fleet of medical services for the elderly (mobile medical network) has been established in major cities in the United States, providing a variety of services such as home medical services and home care services in a midbus for the home-bound elderly in need [13]. It adopts market-oriented operation and professional management, so that the elderly can share service resources and reduce the cost of elderly care services. The UK was the first country to introduce the concept of “smart ageing.” The UK believes that community-based ageing is the most suitable model for ageing in the country. More old people mainly are in the community, including senior housing, day care centres, senior activity centres, and care institutions. [14]. The UK has a high level of enthusiasm for volunteer participation in community-based ageing. Germany is currently one of the most ageing countries in Europe, with 23% of the elderly over 60 years old. The elderly in Germany do not rely on their children for their old age, but mainly rely on themselves and the support of the state and society. In order to cope with the shortage of manpower, Germany is actively developing smart ageing [15]. Japan has the highest level of ageing in the world. In order to cope with the problem of ageing population, Japan attaches great importance to the development of smart ageing as an economic industry. The Housing Authority of Singapore has tested and developed the “Smart Alert System for the Elderly at Home.” The system monitors the lives of the elderly and notifies caregivers in the event of an accident [16].

## 3. Intelligent Device Control

### 3.1. Intelligent Equipment Control

Since its introduction, intelligent device control technology has sparked heated discussions in all sectors of society and has been highly respected by many elderly care institutions in particular as a new type of industrial development driver [17]. Intelligent device control technology not only pushes the development and innovation of intelligent elderly care services to a higher level but also allows the elderly to pursue a more comfortable, safe, and convenient living environment as their living standards continue to improve [18].

The birth of intelligent device control technology is the result of the mutual reaction of the elderly group's pursuit of high-quality physical and mental health and rapidly developing information technology. Intelligent control technology is not only the so-called highly sophisticated technology used in the daily life of the elderly but also control services according to the individual need of the elderly group [19]. Intelligent control technology is the product of a high degree of integration of innovative technologies such as Internet of Things technology, deep neural network algorithms [20], intelligent control technology, and elderly service technology, providing a modern elderly environment with high security, convenience, quality, and comfort for the elderly [21].

### 3.2. Indoor Fall Detection

In this study, it was found that there are two main causes of accidental falls in the elderly population, namely, intrinsic physical factors and extrinsic environmental factors.

A review of the literature on the epidemiology of falls in China revealed that intrinsic factors include dulled senses, reduced vision, slower reflexes, muscle deterioration, reduced balance, and central nervous system disorders, while extrinsic factors include uneven surfaces in the area, poor lighting, cluttered surroundings, and regular use of medications with dizzying side effects. These factors all contribute to the increased likelihood of accidental falls in the elderly population [22]. Reduced balance in older people is a key factor in falling. Factors contributing to unintentional falls in older people are shown in Table 1.

As people walk on their left and right feet, the associated parts of the body work in tandem to maintain balance, and in doing so, they go through a tedious process of musculo-neurotransmission, in which three main mechanisms—perceptual, central, and musculo-organisational—work together. If disturbances in balance occur in the elderly population, such as peripheral neuropathy, vertigo, and visual or muscle strength problems, the risk of accidental falls increases significantly [23].

Falls in older people generally occur when the body's balance mechanisms are accidently disrupted, often within 2 seconds. This is much shorter than normal movements such as squatting, lying down, or standing up. Because the human body falls within a short period of time, the body's centre of gravity is shifted significantly in the direction of the fall, and the fall is accompanied by three specific instantaneous values of acceleration in the *X*, *Y*, and *Z* axes and the angle of tilt in the three axes.

Most studies of accidental falls have used the change in the 3D acceleration and tilt angle values during the fall as a criterion for fall detection. The relationship between the 3D coordinates and the human body is shown in Figure 1.

## 4. Fall Detection Algorithms

The experiment consisted of 8 normal state transitions and 4 indoor fall states. A total of 1080 simulated data were collected, 720 for daily activities and 360 for falls. It was found that placing the integrated sensor at the waist to obtain the acceleration signal of the human body can more accurately reflect the degree of change of the overall movement state, while the more complex transformation of the wrist or arm cannot fully reflect the information of the human posture transformation. Therefore, the optimal position for the sensor was chosen to be the waist and the sensor was fixed directly in front of the volunteer's waist. The required example data are shown in Tables 2 and 3.

When experimenting with the fall detection algorithm, it is important to first sort out the general idea of the entire algorithm process and visualise it using a flowchart. The general framework of the fall detection experiments is shown in Figure 2, with each part of the experiment module described later.

Through the algorithm flowchart, we have a clear understanding of the process of this study on the detection of accidental falls in elderly people, and each step of the algorithm and its principles will be described in detail next.

Noise reduction: based on the fact that the original signal of the sensor is mixed with a large amount of white noise, which must be removed when applied in practical scenarios, this experiment uses wavelet threshold noise reduction to preprocess the original signal [24]. The wavelet threshold noise reduction process is as follows:

1. Wavelet transform of the original signal *f* (*x*) containing noise to obtain the wavelet coefficients *w*(*j*, *k*)
2. Thresholding the coefficient set *w*(*j*, *k*) to obtain an estimated coefficient set *w*(*j*, *k*) such that the difference between *w*(*j*, *k*) and *w*(*j*, *k*)′ is as small as possible
3. The estimated coefficient *w*(*j*, *k*)′ is reconstructed as a wavelet, and the estimated signal *f*(*k*) is the noise-free signal required for the experiment

The angular velocity reflects the tilt of the human body in the room, and the angular velocity of the human body on the three axes during movement can also accurately characterise the change in posture of the elderly. The angular velocities in the three axes are also an accurate representation of the changes in the posture of the elderly. The improved formulae for calculating SMA and angular velocity are shown in equations (1) and (2), where the acceleration values in the *X*, *Y*, and *Z* axes are taken and axis(*t*) is taken as the angular velocity value in the *X*, *Y*, and *Z* axes, respectively.

(1) $$\begin{array}{c} SMA\left(\text{axis}\right)=\overset{n}{\underset{i=1}{\sum }}\left|\text{axis}\left(i\right)\right|, \end{array}$$

(2) $$\begin{array}{c} ta\left(\text{axis}\right)=\int_{t=1}^{\text{timewindow }}w\text{ axis}\left(t\right)\cdot \text{d}t. \end{array}$$

Kernel principal component analysis first maps the original set of feature vectors to a high-dimensional space through a nonlinear transformation and then achieves linear separability in the high-dimensional space to obtain better feature attributes than in the original space [25].

The set of feature vectors {*B*_*n*_}_*i*=1_^*N*^ represents the normalised set of human feature data, where *B*_*n*_ represents the row vector of the *n*th human feature data. For each vector in the set of feature vectors, a suitable nonlinear transformation Φ(*B*_*i*_) : *R*^*m*^⟶*H* *B*_*i*_⟶*B*_*i*_′ is used to map the feature vector *B*_*i*_ into the high-dimensional space *H*. In kernel principal component analysis, the nonlinear transformation Φ(*B*_*i*_) corresponds to a different kernel function *k*(*B*, *B*′). The covariance matrix of the high-dimensional space *H* is shown as follows:

(3) $$\begin{array}{c} \sum =\frac{1}{N}\overset{N}{\underset{n=1}{\sum }}\Phi \left(B_{n}\right)\Phi {\left(B_{n}\right)}^{T}. \end{array}$$

The formula for solving the eigenvalues of the covariance matrix ∑ and its corresponding eigenvectors is shown as follows:

(4) $$\begin{array}{c} \lambda u=\sum u. \end{array}$$

The *i*th eigenvector *u*_*i*_ of the covariance matrix ∑ can be represented by a linear combination of *α*_*n*_^(*i*)^, where *α*_*n*_^(*i*)^ is the summation coefficient, as shown in the following equation:

(5) $$\begin{array}{c} u_{i}=\overset{N}{\underset{n=1}{\sum }}\alpha_{n}^{\left(i\right)}\Phi \left(B_{n}\right). \end{array}$$

Substituting equations (3) and (4) into equation (5) gives

(6) $$\begin{array}{c} \lambda_{i}\overset{N}{\underset{n=1}{\sum }}\alpha_{n}^{\left(i\right)}\Phi \left(B_{n}\right)=\frac{1}{N}\overset{N}{\underset{n=1}{\sum }}\Phi \left(B_{n}\right)\Phi {\left(B_{n}\right)}^{T}\overset{N}{\underset{m=1}{\sum }}\alpha_{m}^{\left(i\right)}\Phi \left(B_{m}\right). \end{array}$$

The inner product operation in the high-dimensional feature space is replaced by a kernel function to obtain

(7) $$\begin{array}{c} k\left(B,B^{\prime }\right)=\Phi {\left(B\right)}^{T}\Phi \left(B^{\prime }\right). \end{array}$$

Multiply both sides of the equal sign in equation (6) by Φ(*B*′)^*T*^ at the same time to obtain

(8) $$\begin{array}{c} \lambda_{i}\overset{N}{\underset{n=1}{\sum }}\alpha_{n}^{\left(i\right)}k\left(B^{\prime },B_{n}\right)=\frac{1}{N}\overset{N}{\underset{n=1}{\sum }}k\left(B^{\prime },B_{n}\right)\overset{N}{\underset{n=1}{\sum }}\alpha_{m}^{\left(i\right)}k\left(B_{n},B_{m}\right). \end{array}$$

According to (8), it is possible to calculate the elements of the kernel matrix as shown in the following equation:

(9) $$\begin{array}{c} K_{mn}=k\left(B_{m},B_{n}\right). \end{array}$$

To make the mean (1/*N*)∑_*i*=1_^*N*^Φ(*B*_*i*_)=0, the kernel matrix *K* in the centralized high-dimensional feature space is also needed.

Unsupervised pretraining: for the data feature of accidental indoor falls by elderly people, this topic uses self-encoders for layer-by-layer unsupervised pretraining to solve the gradient diffusion problem. The hidden layers of the deep neural network are pretrained layer by layer, and the parameters obtained from the pretraining are used as initialisation values for the corresponding parameters of the full algorithm.

To facilitate the computation of feature vector sets, the raw signals including all anomalies and daily behaviour are intercepted as time segments in this experiment. The length of the time slice contains enough information about the elderly action transformation for the computation of the feature vector set and does not produce too long a response delay. The calculation of the components of the feature vector set in this experiment is based on the original signal data population within the time window.

Detection and recognition classifier: based on the efficiency and real-time criteria of the fall anomaly detection algorithm, especially the requirement that the fall algorithm can accurately determine the behavioural characteristics of the elderly, this experiment decided to use a deep neural network based on the back propagation algorithm as the detection and recognition classifier for the whole fall algorithm. The deep neural network classifier designed in this experiment has 2 neurons corresponding to the classification output and a forward fully connected pattern between the layers.

## 5. Assessment of Fall Test Results

Evaluation metrics for determining whether a fall detection algorithm is efficient usually include sensitivity and specificity. In this study, in order to effectively compare the performance of classifiers, it was decided to use an evaluation performance metric commonly used in deep learning and statistics, namely, the error matrix [26]. The error matrix is a standard format for accurate evaluation, and these metrics reflect the performance of the classifier from different aspects. The error matrices are shown in Table 4. Sensitivity refers to the rate at which all fall abnormalities are accurately identified in older people, and specificity refers to the rate at which all normal everyday behaviours are accurately detected in older people.

The experiment was evaluated three times to assess the classification effectiveness of each part of the feature vector group. Using a comparative validation approach, each feature vector group was selected to train the neural network for recognition and classification.

### 5.1. Single-Variable Controlled Experiments

In this experiment, a single-variable control approach was used, i.e., the selected feature vector sets were not dimensionally reduced by kernel principal component analysis and then trained for deep neural network recognition classification, all other conditions being identical. The classification recognition results based on the single-variable control are shown in Table 5. According to the data in the table, the sensitivity of the feature vector group without kernel principal component analysis dimensionality reduction reached 90.32% and the specificity reached 93.48%. However, there is still a significant difference between the training results obtained by the algorithm and the results obtained by the algorithm.

### 5.2. Bivariate Controlled Experiments

This experiment uses a bivariate control approach based on the above to evaluate the effect of kernel principal component analysis down scaling and unsupervised pretraining on the classification of the test set. Each human activity contained 14 coefficient matrices obtained by modelling the preprocessed example data for training the deep neural network and 14 coefficient matrices obtained by the same method for classification tests of fall abnormal and normal behaviour. The recognition classification results are shown in Table 6. The experimental results show that the sensitivity of recognition classification without kernel principal component analysis and unsupervised pretraining can reach about 94.57% and the specificity can reach about 93.32%. This is still a significant difference compared to 99.21% sensitivity and 98.97% specificity of the algorithm. It can be seen that the deep neural network with kernel principal component analysis and unsupervised pretraining is more robust and has better generalization ability.

### 5.3. Identifying Classifier Experiments

The aim of this experiment was to evaluate the effect of different recognition classifiers on the classification of the test set of fall anomalies. The classifiers selected were support vector machines, shallow feedforward neural networks, and deep neural networks. The tilt angle and signal amplitude were combined into a 14-bit feature vector set, and for each human activity, there were 14 coefficient matrices obtained by modelling the coefficient data after data processing, dimensionality reduction, and unsupervised pretraining for training the three classifiers mentioned above, and 14 coefficient matrices obtained by the same method were used for testing the fall detection classifier. The classification results of the different recognition classifiers are shown in Table 7. According to the experimental results, although the classification results of the first two classifiers have reached a high level of accuracy, there is still a significant gap compared to the deep neural network, which has the advantage of balancing sensitivity and specificity that other classifiers do not have.

## 6. Conclusions

In this paper, a fall detection algorithm based on kernel principal component analysis and deep neural networks is proposed to address a series of urgent problems such as the vulnerability of elderly people to fall indoors and the potential for multiple injuries after a fall. The algorithm takes the raw signal from the integrated sensor, acceleration, and body tilt as the feature vectors to be input, and after dimensionality reduction by kernel principal component analysis and unsupervised pretraining by self-encoder, a deep neural network based on backpropagation algorithm is used as the fall detection classifier. Experimental validation on 1080 sample instances of data achieved a sensitivity of 99.21% and specificity of 99.87%.

## Figures and Tables

**Figure 1:** Schematic diagram of the correspondence between 3D coordinates and the human body.

**Figure 2:** General framework of the fall detection experiment.

**Table 1:** Factors contributing to the occurrence of unintentional falls in older people.

Factor type	Fall inducement
Physical internal factors	Sensory retardation, vision loss, slow response, and central nervous system diseases
External environmental factors	Skeletal muscle degeneration, uneven road surface, insufficient light, disordered environment, inappropriate height of bed and chair, and dizziness and weakness caused by taking some drugs

**Table 2:** Simulated data on daily behavioural activities required for the fall algorithm.

Behaviour type	Human body state transformation	Number of experiments
Daily behaviour activity simulation	From standing to sitting	90
	From sitting to standing	90
	From standing to lying down	90
	From lying down to standing	90
	From sitting to lying down	90
	From lying down to sitting up	90
	Stand and turn left	90
	Stand and turn right	90

**Table 3:** Simulated data for accidental fall activity required for the fall algorithm.

Behaviour type	Human body state transition	Number of experiments
Indoor fall anomaly simulation	Fall to the left	90
	Fall to the right	90
	Fall forward	90
	Fall back	90

**Table 4:** Error matrix.

	Positive sample	Negative sample
Correct	Accidental falls	Daily behaviour
Error	False accidental fall	Pseudo-daily behaviour

**Table 5:** Results of fall detection based on single-variable control method.

Data preprocessing	KPCA dimensionality reduction	Unsupervised training	Recognition classifier	Sensitivity (%)	Specificity (%)
Have	Nothing	Have	Deep neural network	96.32	95.48
Have	Have	Have	Deep neural network	99.21	99.87

**Table 6:** Results of fall detection based on bivariate control methods.

Data preprocessing	KPCA dimensionality reduction	Unsupervised training	Recognition classifier	Sensitivity (%)	Specificity (%)
Have	Nothing	Nothing	Deep neural network	94.57	93.32
Have	Have	Have	Deep neural network	99.21	99.87

**Table 7:** Fall detection results for different recognition classifiers.

Data preprocessing	KPCA dimensionality reduction	Unsupervised training	Recognition classifier	Sensitivity (%)	Specificity (%)
Have	Have	Have	Support vector machine	97.36	97.52
Have	Have	Have	Shallow neural network	96.93	95.41
Have	Have	Have	Deep neural network	99.21	99.87

## Data Availability

Analytical permission was not obtained from the data provider because of trade confidentiality.
